This article has been retracted.

# Expression of Functional Anti-p24 scFv 183-H12-5C in HEK293T and Jurkat T Cells

**DOI:** 10.15171/apb.2017.036

**Published:** 2017-06-30

**Authors:** Mohammad Tasyriq Che Omar

**Affiliations:** ^1^Cluster of Oncology and Radiological Sciences, Advanced Medical and Dental Institute, Universiti Sains Malaysia, 13200 Kepala Batas, Pulau Pinang, Malaysia.; ^2^Biology Program, School of Distance Education, Universiti Sains Malaysia, 11800 USM, Pulau Pinang, Malaysia.

**Keywords:** Single-chain variable fragment (scFv), scFv-Fc, HIV-1 Capsid p24 protein, Mammalian-based expression, Intrabody

## Abstract

***Purpose:*** More than half of the diagnostic and therapeutic recombinant protein production depends on mammalian-based expression system. However, the generation of recombinant antibodies remains a challenge in mammalian cells due to the disulfide bond formation and reducing cytoplasm. Therefore, the production of functional recombinant antibodies in target cell line is necessary to be evaluated before used in therapeutic application such intrabodies against HIV-1.

***Methods:*** The work was to test expression of a single-chain variable fragment (scFv) antibody against HIV-1 Capsid p24 protein in a human mammalian-based expression system using HEK293T and Jurkat T cells as a model. Three expression plasmid vectors expressing scFv 183-H12-5C were generated and introduced into HEK293T. Expression of the scFv was analyzed, while ELISA and immunoblotting analysis verified its binding. The evaluation of the recombinant antibody was confirmed by HIV-1 replication and MAGI infectivity assay in Jurkat T cells.

***Results:*** Three plasmid vectors expressing scFv 183-H12-5C was successfully engineered in this study. Recombinant antibodies scFv (~29 kDa) and scFv-Fc (~52 kDa) in the cytoplasm of HEK293T were effectively obtained by transfected the cells with engineered pCDNA3.3-mu-IgGk-scFv 183-H12-5C and pCMX2.5-scFv 183-H12-5C-hIgG1-Fc plasmid vectors respectively. scFv and scFv-Fc are specifically bound recombinant p24, and HIV-1 derived p24 (gag) evaluated by ELISA and Western blot. Jurkat T cells transfected by pCDNA3.3-scFv 183-H12-5C inhibit the replication-competent NL4-3 viral infectivity up to 60%.

***Conclusion:*** Anti-p24 scFv 183-H12-5C antibody generated is suitable to be acted as intrabodies and may serve as a valuable tool for the development of antibody-based biotherapeutics against HIV-1.

## Introduction

The development of smaller antibody fragments, which maintain the antigen affinity of the parental antibody, is preferable for better antibody production. Furthermore, the advance in smaller fragments production is the primary source for the *in vitro* antibody generation systems.^1-3^ The Fv fragment that comprises of variable (V) regions is the smallest antigen-binding fragment that maintains the parental antibodies antigenicity properties. To connect the V regions, a soluble and flexible amino acid peptide linker is applied to a scFv (single chain fragment variable) fragment.^4-6^ Nowadays, two standard formats of recombinant antibodies that are produced in eukaryotes expression system are scFv and Fab that show relevant for the clinical evaluation purposes.^7^ Moreover, a fusion of the Fc domain towards antibody fragments result in regaining effector functions, stability, and avidity.^8,9^

Recombinant antibodies targeting HIV-1 virus proteins have shown a potential in inhibiting the virus replication and infectivity. The recombinant antibodies are acting either as an intracellular antibody (intrabody) or transbody to achieve the requirement effects. Since early 1990 until 2016, four leading groups and few small laboratories had developed eight intrabodies against HIV-1 virus proteins. Marasco group focused on the generation of intrabodies like anti-Tat, anti-gp120, and anti-MA p17.^10-14^ Meanwhile, Pomerantz and colleague worked on the production of anti-Rev, integrase, and reverse transcriptase intrabodies.^15-17^ Designing of anti-CCR5, anti-Vif, and integrase intrabodies is the main focusing by Barbas III and Goncavales group.^18-20^ In our knowledge, there is no works about the establishment of anti-CA p24 from anti-p24 hybridoma cell line and used as intrabodies in inhibiting the HIV-1 virus replication and infectivity. Here, we are the first group reporting the intrabody.

Mammalian cells are predominantly used as expression hosts for heterologous protein production despite being harder to maintain compared to bacteria or yeast. Industrial pharmaceutical showed almost up to 50-60% of approved recombinant proteins and antibodies were produced in mammalian-based cell system.^21^ HEK293T is among several cell lines derived from a human mammalian cell that used for the production of recombinant antibody. Frank Graham established human embryonic kidney 293 (HEK293) cells in 1973 at experiment number 293 by using DNA of Adenovirus 5.^22^ DuBridge and the group then developed a cell line that stably transfected with the simian virus 40 (SV40) large T antigen for use in transient production process.^23^ The cell line allows the episomal propagation thus enhancing the total yield of production process.^24^ The cell line also resists against geneticin (G418) as result of the expression of neomycin phosphotransferase (Neo) selection marker. Therefore, stable transfection with any plasmids containing Neo is not possible with this cell line.^25^ For last ten years, approximately 15% of scientific publications have used HEK cells, and the percentage will expectedly increase in the next decade.^26^

The used of relevant cells in biology assessment is important to mimic the real situation of HIV-1/AIDS progression. Jurkat T cells are human acute lymphoblastic leukemic T cell line that is stably producing human interleukin 2.^27,28^ The cell line derived from Fred Hutchinson Cancer Research Center and had designated as Jurkat-FHCRC. The cells were then subjected for limiting dilution to obtain Jurkat Clone E6-1 that now distributes by ATCC and NIH AIDS Reagent Program companies.^29^ The cells have been popularly used for biology evaluations with nearly 17,000 Pubmed references for Jurkat from late 1980 until 2016. There are about 1,320 Pubmed literatures related with Jurkat and HIV-1 suggesting the model is a gold standard for assessment of HIV-1 replication and infectivity. HIV-1 Tat increased the CD4 receptor expression of Jurkat cells that led susceptibility to HIV-1 virus infection.^30^ In fact, HIV-1 infected CD4^+^T can produce up to 10x10^9^ virions per day in an infected person and bear a half-life of 2.2 days.^31^

In this study, anti-p24 scFv was expressed in the human mammalian-based system, and its functional activity was evaluated with the hope that antibody-based biotherapeutics can be developed as an alternative treatment against HIV-1/AIDS.

## Materials and Methods

### Bacterial strains and culture conditions

The *E. coli strain* DH5α (NEB, #C2987) was used for cloning and plasmid propagation purposes. Bacterial strains were grown aerobically in Luria-Bertani (LB) broth, or on LB agar at 30^o^C, and in the presence of Ampicillin (100 µg mL^-1^). Bacterial strains were stored in glycerol (50%) -supplemented LB broth at -80°C.

### General molecular biology techniques

PCR amplifications of DNA fragments intended for cloning purposes was carried out using Q5® High-Fidelity DNA Polymerase (NEB, #M0491), whereas Taq DNA Polymerase (NEB, #M0273) was used for routine colony PCR. PCR amplified or restricted DNA fragments were purified using NucleoSpin® Gel and PCR Clean-up kit (Macherey-Nagel GmbH & Co, #740609). Plasmid DNA was purified using Wizard® Plus SV Minipreps DNA Purification System (Promega, #A1465). Vector and insert were mixed in 1:3 molar ratios (unless otherwise specified) and ligated in the presence of T4 DNA ligase (NEB, #M0202) at 4^o^C for 18 h. 100 μl of *E.coli* DH5α as competent cells was transformed with 5 μl of vector-insert ligation mix and selected on LB agar plates containing 100 μg/mL ampicillin at 30°C overnight incubation. For colony PCR, at least ten randomly selected bacterial colonies were PCR amplified using a vector -specific and an insert -specific primer. Plasmid DNA was isolated from positive transformants that contained amplicon of expected size by PCR and then verified using DNA restriction.

### Engineering of the scFv expression vectors

#### pCDNA3.3-scFv 183-H12-5C

scFv 183-H12-5C was cloned in pCDNA 3.3_mCherry that was obtained from Derrick Rossi (Addgene plasmid # 26823). To replace mCherry with scFv insert, inverse amplified of pCDNA3.3_mCherry by using pCDNA3.3-*Sfi*I-R1 and pCDNA3.3-*Not*I6H-F1 primers (Table 1) was performed. The process resulted in the removal of mCherry insert and introduction of *Sfi*I (downstream CMV promoter) and *Not*I (upstream TK polyadenylation signal) restriction sites. The resulting PCR amplified vector backbone was reaction cleaned up and sequentially restricted with *Sfi*I and *Not*I following manufacturer’s protocol. A 783 bp of scFv 183-H12-5C DNA sequence was amplified from a pHEN2-scFv 183-H12-5C (46) plasmid using primers scFv 183-H12-5C-*Sfi*I-F and scFv 183-H12-5C-*Not*I-R (Table 1) and cloned the respective gel purified inserts into the pCDNA3.3 at the same sites. The resulting vector was named pCDNA3.3-scFv 183-H12-5C (46) and transformed into *E.coli* DH5α. The positive clones were screened using vector-specific CMV-F and insert-specific scFv 183-H12-5C-R primers (Table 1). The plasmid was also extracted out before verified using *Sfi*I and *Not*I enzymes

#### pCDNA3.3-mu-IgGk-scFv 183-H12-5C

To introduce *BsiW*I and* Sfi*I restriction sites, the plasmid was inverse amplified by using scFv 183-H12-5C-*Sfi*I-F1 and CMV-*Bsi*WI-R1 primers (Table 2). The process resulted in the introduction of *Bsi*WI (downstream CMV promoter) and *Sfi*I (upstream scFv 183-H12-5C) restriction sites. The resulting PCR amplified vector backbone was reaction cleaned up and sequentially restricted with *Bsi*WI and *Sfi*I following manufacturer’s protocol. Mouse IgG kappa chain signal peptide (Table 2) was oligo annealed in the purified vector. The resulting vector was named pCDNA3.3-mu-IgGk-scFv 183-H12-5C (46) and transformed into *E.coli* DH5α. The positive clones were screened using by using vector-specific 6His-A-Seq-R and insert-specific *Bsi*WI-MuIgGk-F primers (Table 2). The plasmid was also extracted out before verified using *Bsi*WI and *Not*I enzymes.

#### pCMX2.5-scFv 183-H12-5C-hIgG1-Fc

scFv 183-H12-5C was cloned in pCMX2.5-hIgG-Fc that was obtained from Micheal Hust (Technische Universität Braunschweig). To allow the cloning of a scFv insert into the vector backbone, the pCMX2.5-hIgG-Fc vector was restricted in SYBR® Safe DNA gel using *Nco*I and *Not*I restriction enzymes following manufacturer’s protocol. This resulted in accessible of *Nco*I (downstream CMV promoter) and *Not*I (upstream hinge-IgG-Fc sequence) restriction sites. The respective gel purified vector was reaction cleaned up. The scFv insert was prepared by restricting pHEN2-scFv 183-H12-5C-6His-myc with *Nco*I and *Not*I and cloned the respective gel purified inserts into the pCMX2.5-hIgG-Fc at the same sites. Both vector and insert were ligated and incubated overnight. The resulting vector was named pCMX2.5-scFv 183-H12-5C-hIgG-Fc and transformed into *E.coli* DH5α. The positive clones were screened using vector-specific CMV-F and insert-specific scFv 183-H12-5C-*Not*I-R primers (Table 3). The plasmid was also extracted out before verified using *Nco*I and *Not*I enzymes.

**Table 1:** Oligonucleotides used for engineering of pcDNA3.3-scFv 183-H12-5C-6His. Restriction enzyme (italic) and its recognition site underline.

**Set**	**Primer name**	**Primer sequence (5'⟶3')**
**For engineering of pcDNA3.3-scFv 183-H12-5C-6His**		
**1**	pcDNA3.3-*Not*I6H-F	AACGGGCGGCCGCACATCATCATCACCATCACTGAAGGGTTCGATCCCTACCGG
	pcDNA3.3-*Sfi*I-R	CCATGGCCGGCTGGGCCGCAGGGTTCGATCCTCTAGAGTCCGG
**2**	scFv 183-H12-5C-*Sfi*I-F	CCTGCGGCCCAGCCGGCCATGGCCCAGGTCCAACTGC
	scFv 183-H12-5C-*Not*I-R	GATGTGCGGCCGCCCGTTTCAGTTCCAGTTTGGTC
**For colony PCR of scFv 183-H12-5C in pCDNA3.3 plasmid backbone**		
**1**	CMV-F	CGCAAATGGGCGGTAGGCGTG
	scFv 183-H12-5C-*Not*I-R	GATGTGCGGCCGCCCGTTTCAGTTCCAGTTTGGTC

**Table 2:** Oligonucleotides used for engineering of pcDNA3.3-mu-IgGk-scFv 183-H12-5C-6His. Restriction enzyme (italic) and its recognition site underline.

**Set**	**Primer name**	**Primer sequence (5'⟶3')**
**For engineering of pcDNA3.3-mu-IgGkappa-scFv 183-H12-5C-6His**		
**1**	scFv 183-H12-5C-*Sfi*I-F1	CCTGCGGCCCAGCCGGCCATGGCCCAGGTCCAACTGC
	CMV-*Bsi*WI-R1	CCATCGTACGTCGATCCTCTAGAGTCCGGAG
**2**	Mu IgG k-F	GTACGATGGAGACAGACACACTCCTGCTATGGGTACTGCTGCTCTGGGTTCCAGGTTCCACTGGTGACGCGGCCCAGC
	Mu IgG k-R	GGGCCGCGTCACCAGTGGAACCTGGAACCCAGAGCAGCAGTACCCATAGCAGGAGTGTGTCTGTCTCCATC
**For colony PCR of murine-IgG kappa-scFv 183-H12-5C in pCDNA3.3 plasmid backbone**		
**1**	*Bsi*WI-MuIgGk-F	CGTACGATGGAGACAGACACACTCCTG
	6His-A-Seq-R	CCTTCAGTGATGGTGATGATGATGTGC

**Table 3:** Oligonucleotides used for verification of pCMX2.5-scFv 183-H12-5C-hIgG1-Fc. Restriction enzyme (italic) and its recognition site underline.

**Set**	**Primer name**	**Primer sequence (5'⟶3')**
**For colony PCR of scFv 183-H12-5C in pCMX2.5 plasmid backbone**		
1	CMV-F	CGCAAATGGGCGGTAGGCGTG
	scFv 183-H12-5C-NotI-R	GATGTGCGGCCGCCCGTTTCAGTTCCAGTTTGGTC

#### Cell line and culture conditions

HEK293T (#CRL-3216) was purchased from American Type Culture Collection (ATCC). Jurkat T Clone E6-1 (#177) was obtained through the NIH AIDS Reagent Program, Division of AIDS, NIAID, NIH. Jurkat T cell line was maintained in RPMI 1640 supplemented with 2mM L-glutamine and 10%FBS at 37°C in a 5% CO_2_ incubator. HEK293T cells were maintained in Dulbecco’s modified Eagle’s medium (DMEM) supplemented with 10% fetal bovine serum (FBS) at 37°C in a 5% CO_2_ incubator.

#### Transient transfection assay 

#### X-tremeGENE HP DNA Transfection

The day before transfection, 293T cells was cultured at 37°C in 5% CO_2_ to a density of about 5×10^5^ cells/ml in 6-well plates in DMEM medium that contained 10% heat-inactivated FBS. The cultures were 80% confluent on the day of transfection. The scFv vector was transfected into 293T cells using the X-tremeGene or calcium phosphate. Briefly, X-tremeGENE HP DNA Transfection Reagent was used to deliver pCDNA3.3-mu-IgGk-scFv 183-H12-5C plasmid into HEK293T cells. HEK293T cells were seeded at a cell density of 5 x 10^5^ cells per plate onto a 60-mm tissue culture dishes in 5 mL DMEM medium containing 10% FBS the day before transfection. 5 μg of pCDNA3.3-mu-IgGk-scFv 183-H12-5C (stock 1mg/mL) plasmid was gently mixed with 500 μL of DMEM-serum free medium in 1.5 mL tube. Ten μL of X-tremeGENE HP DNA Transfection Reagent (2:1) was added directly into diluent without any contact with the wall of the tube. The complex was gently mixed by pipetting up and down. The transfection reagent: DNA complex was incubated for 15 minutes at room temperature. The transfection complex was added to the cells in a dropwise manner, and the cells were incubated for 24 and 48 hours before measuring protein expression in the culture supernatant.

#### Calcium Phosphate Transfection

Calcium Phosphate transfection was used to deliver pCMX2.5-scFv 183-H12-5C-hIgG1-Fc plasmid into HEK293T cells. HEK293T cells were seeded at a cell density of 5 x 10^5^ cells per plate onto a 60-mm tissue culture dishes in 5 mL DMEM medium containing 10% FBS the day before transfection. Next day, medium on cells was changed three hours before beginning transfection. 2 μg of plasmid was gently mixed with 296 μL of filtered deionized water in 4 mL clear round-bottom tube by vortexing on a low setting (1000 rpm for 10 seconds). 37 μL of 2 M calcium chloride was added to the DNA/water mixture and gently mixed by vortexing on a low setting. 300 μL of 2X HBS was added into new clear round bottom tube and the DNA/water/CaCl2 mixture we dropwise added into it and vortexing on a low setting. The tube was incubated at room temperature for 30 minutes. The mixture was mixed and dropwise added to the pre-warmed medium on the cells with gently swirling. The cells were incubated for 16 hours before changed with fresh medium. The culture supernatant was collected after 48, 72 and 96 hours before continuing with purification.

#### Neon Transfection System

For difficult transfected cells such human Jurkat T cell, introducing plasmid into this cell was done by electroporation using Neon Transfection system. The cells were washed with 1X PBS once and diluted to 3x10^6^ cells/30uL in R-Buffer. 0.3x10^6^ cells (10 μL) were gently mixed with pCDNA3.3-scFv 183-H12-5C (3 μg) in a sterile 0.2 mL tube. 10 μL of the mixture that represents 0.2x10^6^ cells and 2 μg plasmids were used for electroporation with parameters; pulse voltage=1300, pulse width=10, and pulse number=3. The transfected cells were maintained at 0.2x10^6^ cells/mL in pre-warmed RPMI 1640 growth medium and incubated at 37°C for 48 hours to allow cells to recover. The cells were used for antiviral assessment.

#### Purification of scFv 183-H12-5C and scFv-Fc 183-H12-5C

The clear supernatant containing soluble scFv 183-H12-5C-6His was filtered through pre-washed (with deionized H_2_O) 0.45 μm membrane (Millipore, #HPWP04700) and diluted 1:1 with equilibrium/wash buffer (50 mM sodium phosphate, 300 mM NaCl, 20 mM imidazole, pH 7.4). The sample was loaded onto a 1 mL HisPur Cobalt Chromatography Cartridge at a flow rate of 1 mL/min. The cartridge was washed with equilibrium/wash buffer until the baseline absorbance at 280 nm was reached. scFv His-tagged was eluted with 20–150 mM imidazole gradient, collected in 1 mL fractions.

The supernatant containing soluble scFv-Fc 183-H12-5C of the transiently transfected cells was applied to Pierce™ Chromatography Cartridges Protein G (Pierce #89926) on an FPLC system (AKTA purifier 900, GE) that had been previously equilibrated with binding buffer (50 mM sodium acetate, pH 5.0). The column was washed with binding buffer, and protein was eluted with a linear imidazole gradient (5-150 mM in 0.1 M glycine, pH 2.5). The eluted fractions were collected in tubes that contained a neutralizing buffer (1 M Tris-HCl, [pH 8.0]), so as to adjust the pH to approximately 7.

Finally, the purified samples (scFv and scFv-Fc 183-H12-5C) were dialyzed against PBS. Dialysis was performed three times with an exchange of fresh PBS in each round. The dialyzed products were lyophilized and reconstituted in deionized H_2_O followed by quantification using Qubit Protein fluorometer. The purity of the eluted antibody fraction was analyzed by SDS-PAGE on 10% gels under reducing conditions. Protein bands were visualized by Coomassie blue staining. After electrophoresis, the proteins in the gel were transferred to a nitrocellulose membrane (GE), which was then blocked with 5% skim milk in TBST (TBS with 0.05% Tween 20). The membrane was incubated with a 1：10,000 dilution of HRP-conjugated goat anti-human IgG (KPL) for 1 h at room temperature and then washed three times with TBST. After that, the immunoreactive bands were visualized using an enhanced chemiluminescence detection system (ECL; Pierce Thermo).

#### Binding activity of scFv 183-H12-5C and scFv-Fc 183H12-5C

Binding activities of scFv and scFv-Fc antibody were determined by western blot and ELISA. For ELISA, serially dilutions of scFv 183-H12-5C-6His (160 nM -10 nM) in coating buffer and 100 µL used to coat individual wells of a 96-well microliter plate. Parental anti-p24 IgG mAbs (183-H12-5C) were used to coat some wells that served as positive control. The plate was incubated overnight at 4^o^C and wells were washed 3X with wash buffer (PBS pH7.4, 0.05% Tween-20). Occupied sites were blocked by incubating wells with 200 µL of blocking buffer (PBS pH7.4, 5% skimmed milk) for two h at 25°C followed by 3X washing with wash buffer before adding the samples. 100 µL of HIV-1 derived p24 (gag) were added to each well, lysed with 25 uL of lysis buffer and incubated at 25°C for two h. The wells were washed and added with 100 µL of 33.33 nM (5µg/mL) of HRP-conjugated secondary anti-p24 mAb (31-90-25) and incubated at 25°C in the dark for 1 hour. The wells were washed and bound antibody detected by adding 100 µL of TMB substrate solution (KPL #52-00-01) for 30 min at 25^o^C in the dark. The color development was stopped by adding 100 µL of 0.5M sulfuric acid and absorbance was measured at 450 nm with a reference wavelength of 670 nm.

Meanwhile, for scFv-Fc 183-H12-5C, two dilutions (1 and 10 ug/mL) of recombinant p24 in coating buffer were used to coat individual wells of a 96-well microliter plate. The plate was incubated overnight at 4°C and wells were washed 3X with wash buffer (PBS pH7.4, 0.05% Tween-20). Occupied sites were blocked by incubating wells with 200 µL of blocking buffer (PBS pH7.4, 5% skimmed milk) for two h at 25°C followed by 3X washing with wash buffer before adding the samples. 100 µL of 1 ug/mL of scFv-Fc 183-H12-5C were added to each well and incubated at 25^o^C for two h. The wells were washed and added with 100 µL of 33.33 nM (5µg/mL) of HRP-conjugated anti-human mAb (KPL) and incubated at 25°C in the dark for 1 hour. The rest steps as mentioned in above.

For Western blot, proteins (recombinant P24 or inactivated HIV whole virus) were transferred to nitrocellulose membrane (GE Healthcare Life Sciences, # RPN82D), blocked with blocking buffer (5% skimmed-milk proteins in TBS-Tween 20), and incubated either with 2 mL of scFv-Fc (1 µg/mL) or mAb-IgG 183-H12-5C (1μg/ml) diluted in 5% skimmed milk TBS-T for 12 h at 4^o^C. Blots were washed 3X with washing buffer (TBS, 0.1% Tween-20) and bound scFv-Fc and mAb were probed using two mL of anti-human IgG-HRP (KPL) and anti-mouse IgG-HRP respectively, diluted 1:20,000 in 5% skimmed milk TBS-T was added and blots incubated at 25°C for one h. Blots were developed by using SuperSignal West Pico reagents after washing 3X with washing buffer.

#### HIV-1 replication analysis

Jurkat T cells (1x10^5^ cell/well) were transfected with 1 μg of pCDNA3.3-scFv 183-H12-5C by Neon Transfection system. After 48 hours, cells were counted and dispensed into 1.5 mL tubes at a cell density of 1x10^5^ cells/tubes in 0.05 mL complete medium (RPMI containing 10% FBS) with 20 μg/mL DEAE-dextran. Cells were infected at a multiplicity of infection (MOI) of 0.1 with replication-competent HIV-1 NL4.3

#### MAGI infectivity assay

MAGI cells were seeded at a cell density of 1 x 10^4^ cells per well onto a 96-well plate in 0.1 mL complete DMEM the day before infection. Next day, the medium was removed and 30 μL viral supernatant diluted in serum-free DMEM containing 20 μg/mL DEAE-dextran (BioBasic, Canada #DB0147) was added to each well. The plate was incubated at 37°C, 5% CO_2_ for two hours and 0.2 mL complete media was added. Cells were incubated at 37°C, 5% CO_2_ for two days. Then, cell supernatants were removed, and 0.2 mL of fixing solution (1% formaldehyde, 0.2% glutaraldehyde in 1X PBS) was added to each well. The plate was incubated at room temperature for exactly 5 minutes. The fixing solution was removed and washed thrice with 0.2 ml 1X PBS (pH7.4). Next, cells were stained with 80 μL staining solutions per well and incubated at 37°C for exactly 50 minutes in the non-CO_2_ incubator. The staining solution was removed and washed thrice with 1X PBS (pH 7.4). Blue foci were counted microscopically using inverted microscope and infection levels were recorded as blue focus units (BFU/well). Background levels of BFU/well were typically <2 in all assays.

## Results

### Engineering of pCDNA3.3 -scFv 183-H12-5C

The inverse PCR of pCDNA3.3 vector resulted in the generation of vector plasmid with 5.5 kb (Figure 1B). Amplification of insert-specific scFv 183-H12-5C from pHEN2-scFv 183-H12-5C (46) plasmid resulted in production of insert with 783 bp (Figure 1B). Twelve colonies were randomly selected using a combination primer set and nine out of twelve were amplified around 850 bp scFv 183-H12-5C-6His (Figure 1C). Three positive colonies were then selected and verified with *Sfi*I and *Not*I restriction enzyme respectively. All clones were successfully restricted by detection of linearized plasmids as showed in Figure 1D.

### Engineering of pCDNA3.3-mu-IgGk-scFv 183-H12-5C

The inverse PCR of pCDNA3.3-scFv 183-H12-5C vector resulted in the generation of vector plasmid with 6.19 kb. Oligo annealing of mouse IgG kappa chain signal peptide resulted in ligation with the purified vector that was verified by amplification of scFv 183-H12-5C-6His with 780 bp from twelve randomly transformed colonies (Figure 2B). Five positive colonies were then selected and further restricted with *Bsi*WI and *Not*I restriction enzyme respectively. Two clones were successfully restricted by detection of ~5.4 kb (pCDNA3.3) and 855 bp amplicons as showed in Figure 2C.

### Engineering of pCMX2.5-scFv 183-H12-5C-hIgG1-Fc

The restriction of pHEN2-scFv 183-H12-5C (46) plasmid vector resulted in generation of scFv 183-H12-5C (insert) with size ~780 bp. The restriction of pCMX2.5-hIgG-Fc plasmid vector resulted in production of plasmid vector with 5711 bp size (Figure 3B). Twenty-four colonies were randomly selected using a combination primer and twenty-one out of twenty-four colonies were amplified around 850 bp scFv 183-H12-5C-6His (Figure 3C). Six positive colonies were then selected and verified with *Nco*I and *Not*I restriction enzymes. All clones were successfully restricted by detection of 5.711kb (pCMX2.5-hIgG-Fc) and 780 bp (scFv 183-H12-5C) as showed in Figure 3D.

**Figure 1:** Engineering and verification of pCDNA3.3-scFv 183-H12-5C vector. Schematic representation of expression vector pCDNA3.3-scFv 183-H12-5C (A). scFv 183-H12-5C gene was amplified from pHEN2-scFv 183-H12-5C, restricted and cloned at *Sfi*I/*Not*I restriction sites in inversely amplification pCDNA3.3 vector (B). Colony PCR used CMV-F/scFv 183-H12-5C *Not*I-R primers; Presence of ~860 bp band in most of the clones suggests the presence of scFv 183-H12-5C in pCDNA3.3-scFv 183-H12-5C plasmid vector (C). Restriction analysis of pCDNA3.3-scFv 183-H12-5C with *Sfi*I/*Not*I (Linearized plasmids) (D).

**Figure 2:** Engineering and verification of pCDNA3.3-mu-IgGk-scFv 183-H12-5C vector. Schematic representation of expression vector pCDNA3.3-mu-IgGk-scFv 183-H12-5C (A). Colony PCR used *Bsi*WI-muIgGk-F/6His-A-seq-R primers; Presence of ~860 bp band in most of the clones suggests the presence of mu-IgGk-scFv 183-H12-5C in pCDNA3.3-mu-IgGk-scFv 183-H12-5C plasmid vector (B). Restriction analysis of pCDNA3.3-mu-IgGk-scFv 183-H12-5C with *BsiW*I/*Not*I (5.4 kb vector backbone + 855 bp insert) (C).

**Figure 3:** Engineering and verification of pCMX2.5-scFv 183-H12-5C-hIgG1-Fc vector. Schematic representation of expression vector pCMX2.5-scFv 183-H12-5C-hIgG-Fc (A). scFv 183-H12-5C gene was restricted from pHEN2-scFv 183-H12-5C used NcoI/NotI enzymes, gel purified and cloned at *Nco*I/*Not*I restriction sites in restricted pCMX2.5-hIgG1-Fc vector (B). Colony PCR used CMV-Seq-F/scFv 183-H12-5C *Not*I-R primers; Presence of ~860 bp band in most of the clones suggests the presence of scFv 183-H12-5C in a pCMX2.5-scFv 183-H12-5C-hIgG1-Fc plasmid vector (C). Restriction analysis of pCMX2.5-scFv 183-H12-5C-hIgG1-Fc with *Nco*I/*Not*I (5.4 kb vector backbone + 855 bp insert) (D).

### Expression of secreted soluble scFv 183-H12-5C and scFv-Fc 183-H12-5C

Since the MBP-scFv 183-H12-5C produced from bacteria efficiently bound the recombinant and wild-type HIV-1 CA p24 (data not shown), it is important to find out if the expression of scFvs in reducing cytoplasm of mammalian cells would also bind to HIV-1 CA p24. Thus, scFv 183-H12-5C was cloned into engineered pCDNA3.3 vector bearing murine IgGk signal that results in the secretion of the soluble scFv in the culture supernatant.

HEK293T cells were transfected with resulting pCDNA3.3-muIgGk-scFv 183-H12-5C vector and culture supernatant containing soluble scFv was collected at the different time point of post-transfection. In control experiments, cells were transfected with parental pCDNA3.3_mCherry vector that expressed similar sized red fluorescent protein (RFP). Fluorescence microscopic analysis showed the transfection efficiency reached 80-90% which suggested the pCDNA3.3 vector regardless the carried gene were suitable to express target protein in HEK293T cells (Figure 4A). Western blot using anti-6His was performed to confirm the expression of soluble scFv 183-12H5C. Using standard protocol, the HEK293T cells transfected with pCDNA3.3-muIgGk-scFv 183-H12-5C vectors produced soluble scFv by detecting the ~29 kDa bands. In contrast, no detection of red fluorescence protein bands was detected since the protein was not tagged with 6His (Figure 4B). The optimizing experiment showed 0.2 μg of pCDNA3.3-muIgGk-scFv 183-H12-5C plasmid is the suitable concentration to transfect HEK293T for expression of secreted-scFv 183-H12-5C. There was no difference between the scFv collected after 24 or 48 hours of post-transfection (Figure 4C and 4D).

**Figure 4:** Expression analysis of secreted scFv 183-H12-5C-6His in HEK293T. HEK293T cells were transfected with 0.2 mg of pCDNA3.3-muIgGk-scFv 183-H12-5C plasmid vector for 48 hours. Expression of control protein was checked by fluorescence microscope (A). SDS-PAGE and Western Blot analysis of secreted scFv 183-H12-5C collected at the different time point of post-transfection (B). Optimization of plasmid concentrations for expression of secreted scFv 183-H12-5C after 24 hours (C) and 48 hours (D) of post-transfection. Error bars show standard deviations calculated from at least two independent experiments each done in duplicate.

The structure of the scFv-Fc 183-H12-5C antibody produced in the reducing environment of HEK293T was analyzed by SDS-PAGE and immunoblot. The scFv-Fc is expected to be demonstrated as a 52 kDa monomer under the reducing conditions as the interaction of CH_3_ domains breaks in the presence of a potent surfactant such as SDS. As shown in Figure 5B, detection of 52 kDa bands confirmed that the scFv-Fc 183-H12-5C was produced in HEK293T cells.

**Figure 5:** Purification of scFv 183-H12-5C and scFv-Fc 183-H12-5C. Twenty milliliters of supernatant fraction diluted 1:1 with binding buffer was applied on HisPur cobalt resin by batch method purification. Following manufacturer’s instruction, scFv 183-H12-5C was eluted with elution buffer. SDS-PAGE analysis and of protein fractions from scFv antibodies purification by batch method (A). 100 milliliters of supernatant fraction diluted 1:1 with binding buffer was applied on Pierce Chromatography Cartridges Protein G, attached to FPLC system (AKTA purifier 900, GE Healthcare). Following manufacturer’s instruction, scFv-Fc 183-H12-5C was eluted with increasing gradient of elution buffer. SDS-PAGE analysis and Western blot analysis of protein fractions from scFv-Fc antibodies purification by FPLC (B).

### Purification of scFv 183-H12-5C and scFv-Fc 183-H12-5C

Since scFvs 183-H12-5C has a hexahistidine tag at its amino terminal. Hence, the recombinant antibodies were purified using HisPur cobalt resin. As shown in Figure 5A, a simple spin-column method led to the recovery of highly purified scFv 183-H12-5C-6His from the supernatant of HEK293T cells. The incubation of the soluble fraction at 4°C for overnight resulted in efficient binding of scFv 183-H12-5C to the resin bed. Washing buffer containing 30 mM of imidazole with six times washing steps was able to remove unbound histidine protein. The bound histidine protein then eluted for four times under acidic condition. Detection of a prominent protein band of approximately 28 kDa under reducing conditions confirmed that the scFv 183-H12-5C-6His was produced in HEK293T cells.

Since scFv-FC 183-H12-5C has a Fc portion at its amino terminal. Hence, the recombinant antibody was purified using Protein G based on Streptococcal protein G bind to human Fc fragments at β-strand 3 and the α-helix. As shown in Figure 5B, purified scFv-Fc 183-H12-5C were obtained from the supernatant of HEK293T cells using a fast protein liquid chromatography method. Almost all of the scFv-Fc 183-12H-5 protein was bound to the Protein G when the supernatant was flowed in protein G cartridge column with flow rate at 1min/mL. 12 mL wash buffer was able to remove the unrelated protein and scFv-Fc was successfully eluted under acidic condition. The purity of the purified scFv-Fc 183-H12-5C was more than 85%, and scFv-Fc was used for all subsequent immunoblot analysis.

### Binding of scFv 183-H12-5C and scFv-Fc 183-H12-5C against recombinant CA p24 and NL4-3 virus

For binding analysis of scFv 183-H12-5C, the recombinant antibody format specifically captured recombinant p24 antigen evaluated by ELISA. Surprisingly, OD values were significantly lower than those obtain from wells coated with parental mAb-IgG 183-H12-5C. As expected, wells coated with BSA did not produce signals (Figure 6A). This result showed that scFv 183-H12-5C generated in reducing environment of mammalian cells specifically reacted with HIV-1-derived p24(gag) protein.

For binding analysis of scFv-Fc 183-H12-5C, the format also specifically captured recombinant p24 antigen in ELISA setting. Interestingly, OD values were significantly no different between wells coated with 10 or 1 μg of recombinant p24. As expected, wells coated with BSA did not produce signals. No signal provided when supernatant of HEK293T cells was used, confirmed the binding is specific by scFv-Fc 183-H12-5C (Figure 6B).

To further confirm the above results, Western blot analysis was performed. Recombinant p24, HIV-1 (NL4.3) whole virus, and Nef (negative control) were electrophoresis resolved in 12% SDS-PAGE. The transferred proteins were washed and blocked before probed with purified scFv-Fc 183-H12-5C and parental antibody mAb-IgG 183-H12-5C. Detection of scFv-Fc 183-H12-5C and mAb-IgG 183-H12-5C was done using HRP-conjugated anti-human and HRP-conjugated anti-mouse. As expected, scFv-Fc 183-H12-5C specifically bind recombinant p24 and viral p24(gag). Interestingly, binding of scFv-Fc 183-H12-5C was stronger than binding of mAb-IgG 31-90-25 that routinely used for immunoblotting analysis (Figure 6C). Together both results of ELISA and Western blot showed that scFv 183-H12-5C and scFv-Fc 183-H12-5C specifically reacted with recombinant p24 and HIV-1-derived p24(gag) protein.

**Figure 6:** Binding analyses of scFv 183-H12-5C and scFv-Fc 183-H12-5C. Wells of ELISA plate were coated with various dilutions of scFv 183-H12-5C or their parental mAbs. 1 µg/mL of recombinant P24 was captured on immobilized scFv or parental mAbs and detected using HRP-conjugated secondary anti-P24 mAbs (31-90-25). Error bars show standard deviations calculated from at least two independent experiments each done in duplicate (A). Wells of ELISA plate were coated with either 1 µg/mL or 10 µg/mL of recombinant P24. 100 µL of 1ug/mL of scFv-Fc 183-H12-5C was added to capture immobilized recombinant p24 and detected using HRP-conjugated secondary anti-Human. Error bars show standard deviations calculated from at least two independent experiments each done in duplicate (B). Recombinant p24 and proteins extracted from HIV-1 virus were electrophoresed and transferred to nitrocellulose membranes. Immunoblotting with mAb-IgG 31-90-25 or scFv-Fc 183-H12-5C antibodies was carried out as described in materials and methods (C).

### scFv 183-H12-5C inhibits the replication-competent NL4-3 viral infectivity in Jurkat CD4+ T cell line.

To determine the effect of the recombinant antibody on HIV-1 viral replication in CD4^+^ T cell, multi-round infectivity assay was performed. T-cell adapted laboratory strain virus such NL4-3 can be propagated in CD4^+^ T cell such Jurkat. The introduction of scFv 183-H12-5C in this cell line by electroporation was hypothesized might affect the HIV viral replication.

Jurkat T cells were transiently transfected with a plasmid expressing scFv 183-H12-5C by the electroporation method. Transfected cells then were infected with molecular clone of NL4-3 and the virus infectivity was monitored by MAGI infectivity assay. At MOI 0.1 with mimicking natural infection process, virus infectivity of Jurkat expressing scFv were reduced by more than 60% from day one until day 4 (Figure 7A and 7B). Together this preliminary data showed that the scFv acted efficiently in inhibition of virus infectivity producing from CD4^+^ T cells.

**Figure 7:** Kinetic analysis of HIV-1 infectivity on Jurkat T cell-scFv 183-H12- 5C infected with HIV-1 NL4-3 virus. To express intracellularly, pCDNA3.3-scFv 183-H12-5C plasmid vector was electroporated into Jurkat T and expressed constitutively under CMV promoter. Transiently expressing scFv 183-H12-5C-6His Jurkat T cells were infected with HIV-1 (NL4.3) at MOI 0.1 and culture supernatants were collected every 24 h and used in MAGI infectivity assay (A). Percentage of HIV-1 inhibition in Jurkat T cell transiently expressing scFv 183-H12-5C (B). The results are representative of three independent experiments each done in duplicate.

## Discussion

Many studies highlighting the use of antibody from commercial hybridoma cell (clone 183-H12-5C) in detecting the HIV-1 capsid protein p24,^32,33^ however until now it has yet to be used for therapeutic purpose of HIV-1/AIDS. With the fact that monoclonal antibodies (mAbs) are highly specific and stable, it becomes an attractive candidate for *in vivo* treatment. Since 1992 once FDA approved the first therapeutic mAb muromonab-CD3, 61 therapeutic mAbs approved by FDA until mid-2016.^34^ Although the number of approved mAbs is encouraging, most of them are limited to target surface antigens that make an intracellular protein such HIV-1 p24 is challenging. The initial part of developing antibody-based biotherapeutic is to test the antigenicity of anti-p24 mAb inside the target cells. However, antibodies do not readily permeate cell membranes, and thus the use of smaller fragment like scFv which easily expressing in the cytoplasm of mammalian is an option. Previously, the monovalent scFv antibody fragment against HIV-1 CA p24 had successfully isolated by phage display technology (data not shown). Expression of the scFv fusion in bacterial cells had shown high potential for production of functional scFv which then being used as detection reagent (data not shown). Although there was one recombinant antibody scFv against HIV-1 CA p24 produced using bacterial-based system had been reported recently, however no antiviral assays were performed using the format in order to validate its function in HIV replication and infectivity.^35^ Here the expression of scFv in the human mammalian-based system was reported and discussed for establishment of antibody-based biotherapeutic against HIV-1.

Recombinant antibodies against HIV-1 p24 were recovered under two different forms: (i) as secreted soluble scFv molecules from the supernatant of pCDNA3.1-mIgG kappa-scFv 183-H12-5C-transfected HEK293T, and (ii) as scFv-Fc in the culture medium of pCMX2.5-hIgG1-scFv 183-H12-5C-Fc-transfected HEK293T. Both forms could be used as biological tools for different purposes such as soluble scFv potentially can be used as an intracellular antibody (intrabody) and scFv-Fc as a detection reagent. Here the study showed that the format expressed in mammalian reducing environment cytoplasm of HEK293T was able to react with recombinant p24 and HIV-1 derived p24 (gag). These findings suggest that the transient expression of scFv 183-H12-5C in HEK293T cells is not toxic to the cells and functionally active. In the case of soluble scFv-Fc 183-H12-5C, the format could serve in conventional diagnostic assays for HIV-1 Gag detection, through specific recognition of the conserved CA p24 epitope. The format can replace the used of full-length IgG clone 183-H12-5C produced from hybridoma system that expensive and time consuming. Indeed, it has been reported that hybridoma cells tend to lose their mAb productivity during long-term cultivation.^36,37^

Furthermore, the constant region (Fc) plays a crucial role in the structural stability of the binding site and antibody conformation. Usually, the human IgG1 hinge region comprises of CH2 and CH3 was molecularly conjugated to the C-terminus of the scFv to generate the bivalent recombinant antibody. The presence of conserved cysteine amino acids in the constant part leads to the formation of disulfide bond which eventually associates the Fc region into dimers. The resulting bivalent recombinant antibody is known as scFv-Fv closely be similar to the structure of intact IgG.^8^ The modifications aimed to increase the affinity of the monovalent scFv- Fc 183-H12-5C against HIV-1 CA p24. The current results are consistent with the result obtained by Ray and group that showed a fusion of Fc region can enhance the activity of anti-GPRV scFv.^38^

Moreover, a fusion of mouse origin scFv with human constant domains (CH2 and CH3) has proven to be beneficial in the clinical setting. Eliminating of the human anti-mouse antibody (HAMA) response can be simply achieved by generating the chimeric antibodies, humanized, and fully human antibodies.^39^ The anti- CEA scFv-Fc (H310A) chimeric antibody exhibited a low incidence of the HAMA response.^40^ These indicated that chimeric antibody is suitable for the assessment in the human clinical stage. Although the present study successfully obtained scFv-Fc 183-H12-5C, the reagent was used only for the detection analysis and not for biology assessment. The used of chimeric scFv-Fc 183-H12-5C in HIV-1 replication inhibition will provide a benefit to the research community. For a reason, the role of scFv-Fc against HIV-1 replication is under investigation.

To act as an intrabody, the scFv must be expressed in the mammalian target cells. The plasmid pCDNA3.3-scFv 183-H12-5C-6His construct was transiently expressed in T cell line and the infectivity of HIV-1 was monitored. The finding revealed that intracellular expression of anti-p24 scFv resulted in the production of functionally active intracellular antibodies (intrabodies) that interacted with incoming HIV capsid and prevented cells from producing the infectious viruses. No genomic integration of the gene of scFv when this type of expression was applied. Since the scFv was expressed episomally, over time the expression of the scFv is lost. Increasing of the infectious virus after day 4 of propagation may reflect from the phenomenon. Despite that, the transient expression is very useful in this study since it directly proved that scFv construct could be expressed well in Jurkat cell and at the same time can react with NL4-3 virus which led to a decrease of infectious virus. The model system used was correlated with the report of effectiveness intrabodies against HIV-1 replication and infectivity.^14,19,20^

Since the transient expression of scFv 183-H12-5C in Jurkat cell showed the potential clinical efficiency, stable expression was preferred for expressing the scFv. The correct integration that allows for scFv expression are small, and for that reason, several rounds of selective pressure in the form antibiotic supplementation needed to be applied for several weeks. However, stable production of scFv 183-H12-5C in Jurkat cells system under controlled of CMV promoter did not work. No expression of the recombinant antibody in developed cell line after selection process although the gene was still presented in the genome of the cells (data not shown). Integration of plasmid into chromosomes from cells grown under selective pressure analyzed by fluorescence in situ hybridization analysis (FISH) demonstrated that the integration constantly happened at a single site irrespective of the transfection method.^41^ This finding suggests that electroporation method was not the cause of the failure in the establishment of stable expressing scFv anti-p24 Jurkat cell line. Currently, to overcome the limitation, engineering the plasmid having another promoter and reporter gene for stably expressing of scFv and transfection efficiency determination in Jurkat cells respectively is undergoing.

## Conclusion

In this work, the mammalian plasmid vectors expressing anti-p24 scFv were successfully engineered. ScFv and scFv-Fc were specifically expressed in a human mammalian-based expression system. The purified scFv and scFv-Fc showed good binding activity and specificity towards recombinant p24 and HIV-1 derived p24 (gag). Intracellular expression in relevant cells also demonstrated the effectiveness of inhibiting HIV-1 replication and infectivity. The antibody could be used as candidates for the development of antibody-based biotherapeutics against HIV-1/AIDS.

## Acknowledgments

Cluster of Oncology and Radiological Sciences, AMDI, USM provided the facilities that were used for the experiments. Mohammad Tasyriq Che Omar was sponsored by the ASTS (Academic Staff Training Scheme USM) (KS4049) and Ministry of Higher Education (MOHE) (KPT860818025037) scholarships during the study.

## Ethical Issues

Not applicable.

## Conflict of Interest

The author declare that there is no conflict of interests regarding the publication of this article.
